# Machine Learning for Healthcare Wearable Devices: The Big Picture

**DOI:** 10.1155/2022/4653923

**Published:** 2022-04-18

**Authors:** Farida Sabry, Tamer Eltaras, Wadha Labda, Khawla Alzoubi, Qutaibah Malluhi

**Affiliations:** ^1^Computer Science and Engineering Department, Faculty of Engineering, Qatar University, Doha, Qatar; ^2^Engineering Technology Department, Community College of Qatar, Doha, Qatar

## Abstract

Using artificial intelligence and machine learning techniques in healthcare applications has been actively researched over the last few years. It holds promising opportunities as it is used to track human activities and vital signs using wearable devices and assist in diseases' diagnosis, and it can play a great role in elderly care and patient's health monitoring and diagnostics. With the great technological advances in medical sensors and miniaturization of electronic chips in the recent five years, more applications are being researched and developed for wearable devices. Despite the remarkable growth of using smart watches and other wearable devices, a few of these massive research efforts for machine learning applications have found their way to market. In this study, a review of the different areas of the recent machine learning research for healthcare wearable devices is presented. Different challenges facing machine learning applications on wearable devices are discussed. Potential solutions from the literature are presented, and areas open for improvement and further research are highlighted.

## 1. Introduction

The last few years have witnessed great advances in wearable technologies. Wearable devices include any device that can be worn by humans such as wristwatches, glasses, chest straps, rings, and prosthetic sockets. Wearable devices belong to the Internet of medical things (IoMT), together with the implantable, ambient, and stationary devices used in hospitals. These devices are typically connected to a network and communicate remotely with mobile devices as shown in Figure 1.

Wearable devices may include different types of sensors to continuously monitor various human signals, e.g., temperature sensors, accelerometers, optical sensors, and biometric sensors. Although the readings of some of these sensors are not yet as accurate as stationary devices in hospitals, they are sometimes considered acceptable [1, 2], depending on the application.

Sensors in IoMT devices and human interaction with these devices are considered a big source of data from which features can be extracted for machine learning (ML) algorithms to detect and learn useful patterns. This can be very useful in many healthcare and elderly care applications such as activity detection for health state assessment, fall detection, stress detection, fitness tracking, vital signs monitoring, and diseases' diagnosis. Using machine learning techniques to learn from human body signals, recorded by wearable devices, has been an active research area in the last decade with a lot of published research studies. Despite this huge research effort and the remarkable growth in using wearable devices, especially smart watches, few machine learning applications for wearable devices have found their way into the market.

Examples include irregular rhythm notification feature [3] in Apple Watch, which won U.S. Food and Drug Administration (FDA) approval with a long list of warnings and precautions in 2018 (https://www.accessdata.fda.gov/cdrh_docs/reviews/DEN180044.pdf), and Eko's heart murmur detection algorithm, which has been recently published [4], which is not really for a personal wearable device but an electronic stethoscope. Additionally, some of the wearable devices that were used for monitoring, which were surveyed in [5], are no longer available in the market. Practical and reliable use of machine learning techniques in the domain of wearable devices is still facing many challenges.

Several review papers have discussed some challenges for wearable devices. In a survey paper published in 2012 [6], the authors focused on some features of wearable devices and their types such as diseases that can be monitored, research prototypes, and challenges such as system efficiency, user perception, cost, social inclusion, and ethical issues. In [5], the authors provided a survey of commercially available wearable devices at that time (2017). They focused on communication security issues, power efficiency, and wearable computing. Neither of the surveys focused on the challenges facing machine learning applications for healthcare wearable devices specifically.

In this study, we review recent applied machine learning research for wearable devices. We identify many challenges facing machine learning applications on wearable devices from design to deployment, such as different deployment alternatives, storage, power consumption, user acceptance, reliability, communication, security, and privacy. We discuss security and privacy both from the data and the model perspectives listing potential solutions to keep subjects' personal data from wearable devices private and secure. Additionally, we review the different privacy-preserving techniques used for machine learning training and inference and discuss their applicability to the model of wearable device usage shown in Figure 1.

The review includes the recent research papers in the field of wearable devices that have been published from 2017 to December 2021 to answer the following questions:

1. What are the healthcare machine learning tasks that have been researched in the literature, the body signals, and techniques used in these tasks?
2. What are the challenges facing machine learning for healthcare wearable devices?
3. What are the possible solutions for these challenges in literature?

Thus, the main focus of this study was to identify the challenges of developing machine learning applications for healthcare wearable devices and alternative solutions found in the literature. Different categories of recent healthcare machine learning research are reviewed while spotting the challenges and highlighting potential research areas and applications that need further investigation.

The rest of the review is organized as follows. In the next section, the necessary background for IoMT and the different human body signals used in wearable devices research are presented. Moreover, applications for machine learning in IoMT are reviewed and categorized referencing some of the recent research work published in each area. In Section 3, different challenges facing machine learning research for wearable devices are reviewed, relevant privacy and security aspects for machine learning applications in IoMT are discussed, and possible solutions in literature are presented. In Section 4, we discuss these solutions, their applicability, and their shortcomings. Additionally, we highlight the main research gaps we perceived in the domain. Finally, the study conclusions are provided in Section 5.

## 2. Wearable Devices and Machine Learning

The wearable device domain is being actively researched for the sake of enhancing ease of use, comfort, and noninvasiveness of monitoring physiological vital signs and sometimes psychological or emotional state, which can be detected by analyzing data from different sensors. Following the tremendous technological advances in the design of system on chip (SoC), the development and use of wearable devices have remarkably achieved high growth rates in the last few years. The wearable device market size was valued at USD 32.63 billion in 2019 and is expected to expand at high rates in the next few years according to the wearable technology market industry report by Grand View Research (https://www.grandviewresearch.com/industry-analysis/wearable-technology-market).

The number of globally connected wearable devices is about to reach 1 billion according to Statista (https://www.statista.com/statistics/487291/global-connected-wearable-devices/). Examples of wearable devices are smart watches, armbands, chest straps, shoes, helmets, glasses, lenses, rings, patches, textiles, and hearing aids [6].

Despite this grand growth, there is still a great need for ongoing research in this area for enhancing the accuracy of these devices, using different body signals for new application areas, and dealing effectively with the complexity of the human body.

### 2.1. Wearable Device's Signals Used in Learning

The human body can be seen in an abstract way as a group of systems (circulatory system, nervous system, respiratory system, digestive system, etc.). It receives a group of inputs and releases a set of outputs as shown in Figure 2. Inputs include the inhaled air, water, food, visual input for all the scenes and objects seen during the day, auditory input for all sounds and voices heard, sensory inputs for the things touched, and olfactory input for things smelled during the day. Outputs include the exhaled air, excretions such as urine, feces, and sweat, skin moisture, body temperature, blood in case of injuries and laboratory tests, energy released by the human in terms of body movements, or performing mental activities and voice output, which can be normal speech, singing, or shouting. Analysis of the inputs and outputs can, to some extent, predict the health state of a person, diagnose possible diseases/disorders, and assist with therapeutic suggestions. These inputs and outputs need to be monitored by wearable devices worn during the day.

Wearable devices include any device mounted on the body and can capture noninvasive signals from the human body through the use of different types of sensors. There are numerous well-known signals and signs that are read from the human body in literature to identify the vital signs and other information about the health or mental state of the subject. Examples of these sensors include skin temperature sensor used in [7, 8] and electrodermal activity (EDA) sensor or sometimes known as galvanic skin response (GSR) sensor used on the skin to record the skin conductance that varies with the sympathetic state of the subject [2]. Other examples include an electrocardiogram (ECG) sensor to capture electrical changes in the skin corresponding to heartbeats used in [9–12]. To capture features of the electrical activity of the brain and the health of muscles and the nerve cells, electroencephalogram (EEG) and electromyography (EMG) sensors are used [13–19]. Blood volume pulse (BVP) can be captured using an optical photoplethysmography (PPG) sensor to estimate heart rate and heart rate variation as in [1, 20–22]. PPG sensor [23] is also used to give an approximation for the oxygen saturation in blood (*SpO*_2_) as in [22, 24]. Accelerometers, gyroscopes, and magnetometers are often used in a wide variety of applications to capture or recognize body movement and activities, which can tell a lot about the health and the lifestyle of the person [1, 25–39].

Other signals that have been used sparingly in literature include electrogastrogram (EGG), which records the electrical activity of the stomach [40], and electrooculogram (EOG), which is generated by eye movements and can be measured with electrodes placed around the eye [41]. Sensory and especially olfactory inputs are challenging to model, but it was observed that the human body has different autonomic responses to different odors, which can be analyzed through the GSR and ECG signals [42]. These inputs can be used in applications including personalized treatments based on odors and foods for neuropsychiatric and eating disorders. Some other inputs may need visual monitoring.  Figure 3 summarizes the different sensors used in the literature for different machine learning healthcare tasks. Features are extracted from these signals to learn a model for either classification or regression of a certain variable. Some literature studies use statistical values such as mean, minimum, maximum, mode, variance, standard deviation, entropy, and kurtosis. However, it is often hard to interpret how some of these statistical features affect the classification or the outcome variable. Additionally, model's accuracy is usually negatively affected by adding more irrelevant features as more is not always better, and domain-specific features that are expressive achieve better performance [43]. Estimating heart rate and breathing rate as features from the PPG signal, change in acceleration magnitude, jerk of motion, and transient changes in skin resistance for seizure detection are examples of domain-specific features. Some applications are concerned with changes happening over a long time period, and some are concerned with transient changes due to certain events such as fall detection and emotion recognition.

### 2.2. Machine Learning for Wearable Devices

Machine learning involves getting wearable devices to act/take decisions without explicit programming for a specific scenario through learning from past experiences. As it is well known, machine learning is usually classified as either supervised, unsupervised, semi-supervised, or reinforced according to the type of the available training data. Learning from past experiences is encoded in terms of data examples that can be either labeled or unlabeled. The target variable for labeled data can be categorical or numerical. Among the tasks that involve machine learning are classification in case of the categorical target output variable, regression in case of numerical labels, and clustering for unlabeled data. Most machine learning research for wearable devices belongs to the classification tasks, some are for clustering [44–46], and few can be tackled as regression problems [43].

Applied research to explore applying machine learning techniques using the body signals discussed in the last subsection for health monitoring, elderly care, and fitness tracking has been growing over the last decade. Among the areas that got researchers' attention are fall detection, seizure detection, vital sign monitoring and prediction [47], and activity recognition for fitness tracking or identifying human daily activities. Additionally, wearable devices have been researched for their use in stress detection and detection of heart rate arrhythmia and rehabilitation tasks. Tables 1–3 show the different areas and a sample of the most recent research work done in each area. The table also shows the machine learning technique(s), sensor(s), and dataset(s) used in each study.

#### 2.2.1. Fall Detection

Three categories of fall detection research efforts can be identified in the literature based on the used technology: (1) wearable devices that use accelerometers and magnetometers, (2) ambient devices such as floor sensors and pressure sensors, and (3) vision-based devices that use monitoring cameras [77].

In [50], the authors reported an accuracy of 99.80% using KNN classifier and 96.82% for falling activity recognition using the random forest classifier. Using tri-axial accelerometer devices [27], KNN, SVM, ANN, and RF classifiers were tested to get a mean average accuracy ranging from 48% to 98% depending on the classifier's task. Some tasks involved distinguishing fall samples from daily activities' samples. Other tasks were to distinguish between different fall samples or different daily activities. The results showed that the classification results on raw data are better than depending solely on the magnitude as feature vector. On the contrary, the magnitude performs better than raw data in the case of subject-independent evaluation. It was easier to distinguish between falls and no falls and subject-independent evaluation testing showed that the classifier performance strongly depends on the subject data. The authors in [78] show the effect of using an optimization technique to increase the accuracy of an SVM classification model.

While the reported accuracy in most of the research done for fall detection is above 90% [28–30], the practicality of these techniques is still questionable as the experiments were done in a controlled environment with a limited number of participants and have the limitation of a high false alarm rate [77]. Another study to simulate fall data [31] was done to generate forward and syncope accelerometer data to form a larger dataset for fall detection training.

#### 2.2.2. Activity Recognition

Activity recognition enables health professionals to get information about a patient's ability (or inability) to perform activities of daily living (ADLs) as a measurement of their health status. Human activity recognition has been researched using convolutional neural networks by the authors in [25], and an accuracy of approximately 96% and 94% was achieved for the UCI-HAR dataset and their study dataset. However, the accuracy of machine learning algorithms for activity recognition for human subjects greatly drops whenever a context of different data distribution compared with that of the training data is confronted [53]. Personalized exercises may be inadequate to be directly used as training data for another subject so the authors in [53] applied a cross-subject transfer learning algorithm that can link source and target signals through the construction of manifolds at the feature level. Another way to approach this problem is to build a personalized model for each subject, and this approach was investigated by the authors in [26] as they see that people perform activities in different ways and that general models may average out important individual characteristics, besides that personalized models can learn from much fewer data and guarantee better privacy for data collected from accelerometers and gyroscopes in wearable devices. Earable (ear-worn) devices can also be used for human activity recognition. They were found to have a superior signal-to-noise ratio under the influence of motion artifacts, and they are less susceptible to acoustic environment noise [79].

Eating activity monitoring, sometimes also referred to as automated dietary monitoring (ADM), is essential for patients' diet assessment and following up with taking medication [33] for elderly people by monitoring taking a pill activity. This is considered an activity recognition task, but it is added to a separate category “Eating Monitoring” in Table 1. In [37], the authors proposed a proximity-based active learning on accelerometer data obtained from a wristband wearable device, which is a novel proximity-based model to recognize eating gestures. In [36], the author assessed using an EMG sensor and contact microphone behind the ear near the jaw to record chewing sounds and detect eating activities. They used 8 features extracted for a 3-second window size for eating detection of crunchy and soft food. A study for eating episode recognition [55] used two IMUs, with one put on ear and the other one on the upper back, and they trained a random forest with the sensors' data and labels. Another study [56] used features from inertial sensor data placed on the downside of the lower jaw to detect eating episodes. A review of the research done until 2019 in the field of eating detection comparing different studies in terms of the used sensors, methods for collecting the data, and evaluation metrics was discussed in [80]. The authors pointed out that most of the studies included accelerometer data from a wrist-worn device for accessibility and ease of use, and they mentioned that the implementation of novel methods for naturally acquiring ground truth remains a challenge. A similar approach can be used for drinking episode detection [81] and smoking cigarette detection [82].

Fitness tracking is another application that can also be considered as an activity recognition task. In [38], the authors were able to identify jogging periods using accelerometers and they concluded that there is no significant benefit from using accelerometers on both hip and ankle locations over using only one accelerometer. Segmentation of exercise and non-exercise periods and recognizing which exercise is being performed were investigated in [57].

#### 2.2.3. Stress Detection

A survey for stress detection using different signals such as heart rate (HR), blood volume pressure (BVP), inter-beat interval (IBI), electrodermal activity (EDA), temperature data, and behavioral features was conducted in [20]. The authors found that the most distinctive features for detecting stress are EDA and HR. Remote monitoring of child safety through stress patterns was tackled in [83]. Detecting stress and anxiety in children with autism spectrum disorder (ASD) was investigated in [58]. The authors in [24] studied stress detection using a neural network for metabolic syndrome patients as the increase in stress may result in chronic symptoms.

Other mental disorders such as depression, anxiety, and bipolar disorder [84] have also been studied in the literature [85] using features from biosignals, eye sensors, microphone, camera, or interactions with smartphone to assess social behaviors.

#### 2.2.4. Arrhythmia Detection

Heart rate tracking could be noticeably seen in some commercial wristband and smart watches. The detection of irregular heartbeats (arrhythmia) is a relatively recent goal for commercial wearables. Fast heartbeats (>rbin100 bpm) are called tachycardia, while slow heartbeats (< 60 bpm) are called bradycardia. Atrial fibrillation is one type of arrhythmia that involves the rapid and irregular beating of the atrial chambers of the heart. Apple conducted a clinical study to detect atrial fibrillation [3] in 419,297 participants using PPG sensors in Apple wrist watch patches, but they used non-machine learning algorithm based on a proprietary threshold analyzed from data for the degree of dispersion of inter-peak intervals to determine irregularity. After a monitoring period and analyzing the results, participants with detected irregularities were notified to do ambulatory ECG monitoring using ECG patches, of which only 34% responded (450 participants). Similar to the clinical study done by Apple [3] to detect atrial fibrillation, Huawei and Fitbit have recently launched their atrial fibrillation study in mid-2020 (https://cardiacrhythmnews.com/wearables-devices-the-new-frontier-in-arrhythmia-management/).

The authors in [59] used the SVM model to identify the raw heartbeats. Then, with an unsupervised dynamic time warping (DTW)-based learning approach using the K-medoids clustering method, the distorted heartbeats are identified and purified. SVM and bagging trees have been used in [11] to detect atrial fibrillation from features from ECG signals.

In [10], the PPG signal was alternatively used. It was recorded for patients with atrial fibrillation using both a conventional oximeter and a cardiotracker ring, which generated comparable results. A convolutional neural network achieved better results when compared to different SVM variants. A worst case accuracy of 94.7% was achieved for 10-second recording periods. Although PPG signals have limitations such as noise introduced by motion artifacts, the authors concluded that the ring PPG-based wearable has good diagnostic performance for atrial fibrillation and can replace ECG-based detection. They also mentioned that considering longer periods for PPG signals may affect the performance due to false positives with atrial tachyarrhythmia episodes. A deep learning model has also been used in [60] but with the best accuracy of 89% achieved learning from both ECG and PPG sensor data.

#### 2.2.5. Seizure Detection

Epilepsy is a neurological disorder that affects the central nervous system, causing seizures or periods of unusual behavior such as twitching in legs and arms and sometimes loss of consciousness. Detecting seizures is important to help the patient get help when needed by alarming a caregiver. Different types of seizures and wearable devices for detecting seizures are reviewed in [86]. The study in [63] included the highest number of participants (135) and used Embrace Empatica Watch [64] with an accelerometer and EDA sensors.

Forecasting seizures can also be useful to alarm the patient to rest and take protective measures. Seizure forecasting has been investigated in [8] using deep learning on multimodal wristband sensor data from 69 patients with epilepsy (total duration >rbin 2,311 hours, 452 seizures). In [62], the authors investigated the use of support vector machine (SVM), random forest (RF), naive Bayes (NB), K-nearest neighbor (KNN), and neural network (NN) to diagnose an epileptic seizure based on EEG sampled dataset available at the UCI machine learning repository. Similarly, the authors in [64, 65] have used both EDA and accelerometer data for detecting seizures but with different datasets and techniques.

#### 2.2.6. Rehabilitation Tasks

Rehabilitation tasks involve tasks to improve abilities needed for daily life, which may be physical or mental abilities that have been lost or impaired due to injury, underlying disease, genetic disorders, or birth defect. One example for a rehabilitation task is foot strike angle prediction, which was studied in [69], which can help in the coaching of running movements and consumer-based shoe prescription. Different machine learning techniques were compared, and random forest achieved the best accuracy of 94.1%.

Linear discriminant analysis (LDA) was used in [87] to classify each subject as a normal or abnormal gait pattern. The authors used real-time acoustic feedback (RTAF) to support the subjects when they are performing the tasks during the rehabilitation session, so that they are able to adjust their motion pattern to the acoustic feedback. Support vector regression (SVR) models yielded excellent intraclass correlation coefficients (ICC) in the gait parameters (stride length, stride velocity, and foot clearance) analyzed in [68] for both walking and running exercises. Similarly, the authors in [67] investigated the same problem on a different dataset using the K-means clustering, SVM, and artificial neural network (ANN).

#### 2.2.7. Hydration Monitoring

Hydration monitoring to detect dehydration is another problem being researched for its importance, especially for athletes, battlefield soldiers, workers in hot conditions, and elderly people who are not able to communicate their need for water. There is an ongoing progress in the development of biochemical sensors that can measure the concentration of different electrolytes in sweat and hence determine the hydration state [88]. Side by side, machine learning research studies try to learn from other different body signals to detect dehydration based on the effect of cognitive stress triggered by dehydration on the autonomic reactions of the body as the work done in [21, 70, 71]. In [71], the authors used heart rate variability (HRV) parameters: RR interval of the ECG signal, standard deviation of RR interval (SDRR), and root mean sum of squares of differences between adjacent RR intervals (RMSSD), from the ECG signal as features with labels at rest, post-exercise, and post-hydration to detect dehydration. The authors in [21] used EDA and other heart rate variability parameters extracted from PPG signal for mild dehydration identification. The authors in [43] used multimodal sources of features from different sensors to predict the last drinking time of the user, which would ease collection of data and provide ways for personalization on-device.

#### 2.2.8. Emotion Recognition

Emotional state monitoring for construction workers in a real worksite using a wearable EEG sensor [15] was classified as positive (e.g., excitement, happiness, contentment, or satisfaction) or negative (e.g., fear, anger, frustration, or depression) based on measuring the EEG valence level and cortisol biochemical response as a reliable marker tested from saliva samples after each task. This can better be performed using machine learning techniques to replace the cumbersome cortisol testing. Considering fear emotional state, fear level classification using different machine learning techniques (KNN, RF, LDA, SVM, and deep learning) has been researched in [89] depending on features extracted from EEG, GSR, HR, and subjective unit of distress (SUD) values in a virtual reality therapy setting. Using EEG raw data, the authors in [16] introduced using a liquid state model (LSM) for training to predict valence, arousal, and liking levels at different durations of the EEG input signal.

#### 2.2.9. Sleep Monitoring

For sleep monitoring and sleep quality assessment, detecting different sleep states (awake, rapid eye movement (REM) sleep stage, and non-REM stages) is a requirement. Classification of sleep episodes has been studied in [32], where a random forest model was used to detect different sleep-wake states with an F1 score of 73.93% after being trained with the data from accelerometers on the wrists of 134 subjects.

Sleep monitoring applications such as detection of sleep apnea episodes have been studied in [1]. Sleep apnea is a problem accompanied by increased cardiovascular risk and decrease in the quality of life. The authors compared auto-correlated wave detection with an adaptive threshold (ACAT) for both electrocardiogram (ECG) data and PPG sensor data to detect the cyclic variation of heart rate (CVHR). The classifier was able to discriminate sleep apnea episodes from non-apnea episodes with 82% sensitivity, 89% specificity, and 85% accuracy depending on PPG signals.

Electrodermal activity, accelerometer data, heart rate variability, and blood volume pressure during sleep have been used in [7] using wearable Empatica E4 smart watch for early detection of migraine from the quality of sleep to enable early alarms to take preventive medication. They achieved a balanced accuracy of over 84% for detecting migraine attacks using quadratic discriminant analysis as a classifier. Another dataset is published in [90] that can be used for sleep stage prediction for which accelerometer and heart rate data were collected from Apple Watch, while the subjects underwent polysomnography during night sleep and it was used for sleep-wake classification in [91] using ANN with accuracy 90%.

- Disease diagnosis artificial intelligence research has been in health care and medical diagnosis of diseases for a long time ago. Starting from expert systems in the 50 s of the last century, continuous efforts have been going on in this field until recently applying deep learning techniques for improved diagnosis of diseases [92]. Examples include lung cancer diagnosis based on CT scans and diagnosis of skin conditions through scanning skin images, which has recently been announced by Google [93]. The use of artificial intelligence and machine learning techniques through wearable devices for initial assisting diagnosis and detection of symptoms is foreseen to be the upcoming future, especially in the COVID-19 pandemic circumstances we are passing through and the quarantine protective requirements imposed in most of the countries.

With the onset of the COVID-19 pandemic, the authors in [76] proposed a protocol for using a mobile health platform to analyze the biosignals recorded by Everion wearable (skin temperature, respiratory rate, blood pressure, pulse rate, blood oxygen saturation, and daily activities), together with a recording for the cough for early detection of COVID patients. For the limited places for patients to receive hospital care, which was observed by the spread of COVID-19 in some countries, the researchers in [22] used machine learning-based analytic systems to detect early signs of clinical deterioration to schedule and guarantee resources' optimization. They also used Everion biosensor to record many physiology parameters such as heart rate, heart rate variability, respiration rate, oxygen saturation, blood pulse, skin temperature, and actigraphy to monitor mild COVID-19 cases and predict clinical deterioration accordingly. Hypertension diagnosis has also been studied in [75] using deep learning for continuous monitoring of blood pressure depending on one-channel ECG and PPG signal that can be obtained from a wearable device.

The use of electronic monitoring devices for asthma has been reviewed in [94]. The authors suggested that clinicians should evaluate asthma management applications to ensure high-quality and evidenced-based information before patients use them as current studies only analyzed asthma patients according to their sleep quality and physical activity measures.

In [95], multiple features of motion and dexterity and sleep measures were collected using IMU sensors on the chest, wrist, and ankle to correlate these measures with measures of neurological disability in multiple sclerosis.

As can be seen from Tables 1–3 and the review in this subsection, no single model can be chosen for every problem as it depends on the dataset size, the features extracted, and the problem being learned. It is very difficult to compare different techniques and the results reported in the research studies as they use different datasets, rely on different features, and solve different problems with multiple experiments. In Figure 4, a box plot is shown for the range of values reported for accuracy of classification models in research studies cited in Tables 1–3 under 5 group models (KNN, SVM, logistic regression, tree-based models (random forest, decision trees, extremely randomized trees), and deep learning (DNN, MLP, LSTM, CNN)). It can be seen that the best median average accuracy achieved is for using deep learning. Logistic regression, SVM, and tree-based models follow deep learning with very close values. All models are away from perfect classification, but some are useful and there is a room for improvement over all tasks using larger datasets, extracting more meaningful features, and modeling for personalization as body signals vary according to each person lifestyle, weight, height, and activity level.

### 2.3. Datasets

PhysioNet (https://www.physionet.org/about/database/) is a big database that offers large collections of physiological and clinical data and related open-source software for research purposes in many areas such as sleep apnea detection, arrhythmia recognition, stress detection, and human activity recognition. It was established by the National Institutes of Health (NIH) and is maintained by MIT Laboratory for Computational Physiology.

There are many other datasets available for human activity recognition and fall detection that are mentioned in [27]. MobiAct [48] (57 subjects/9 ADLs and 4 fall types) is the largest of them in terms of the number of subjects and is suitable for both fall detection and human activity recognition tasks. It is available upon request for research purposes. UCI-HAR dataset [96] provided by the University of California Irvine is the most famous and cited dataset in the domain of human activity recognition. They recorded the 3-axis accelerometer data and 3-axis gyroscope angular velocity time series at 50 Hz for 30 subjects while doing 6 activities (WALKING, WALKING_UPSTAIRS, WALKING_DOWNSTAIRS, SITTING, STANDING, and LAYING) using smartphones banded on the waist.

Friedrich-Alexander-University offers many movement analysis datasets (https://www.mad.tf.fau.de/research/activitynet/) such as daily life activities, step activities, cyclic activities, gait analysis datasets, and energy expenditure estimation. A dataset of 3D accelerometer data specifically for eating activity recognition for 20 participants in laboratory setting and 7 participants in free-living conditions is made available for research purposes by the authors of [56].

A recent real-life human activity dataset was published by the University of A Coruna [97]. They recorded about 189 hours of measurements from the accelerometer, gyroscope, magnetometer, and GPS of smartphones for 19 different subjects with no restriction for mobile position. The data have four labels that define different activities (inactive for not carrying the mobile phone, active for carrying the mobile phone and moving (making dinner, being in a concert, etc.), walking for moving to a specific place whether jogging or running, and driving for moving in a car, bus, truck, etc.).

Sleep Data (https://sleepdata.org/datasets) have large collections of de-identified physiological signals and clinical data elements that are offered by the National Sleep Research Resource (NSRR) to help in sleep monitoring research. Some of these signals can be obtained through wearable devices using different sensors' types.

RecoFit [57] contains accelerometer and gyroscope recordings from over 200 participants performing various gym exercises.

The seizure gauge dataset (https://www.epilepsyecosystem.org/my-seizure-gauge-1) records long-term physiological signals such as EMG, PPG, EEG, ECG, accelerometer signals, BVP, EDA, and temperature from different people with epilepsy using three different wearable devices.

iRhythm arrhythmia detection public test dataset (https://irhythm.github.io/cardiol_test_set/) is a dataset used in [9] for testing a model used for arrhythmia classification for 336 records of 30 s strips single-lead ECGs captured at 200 Hz from 328 patients who used a single-lead ambulatory ECG monitoring patch. Each record is annotated by a consensus label obtained by a committee of three cardiologists.

A database for emotion analysis using EEG signals (https://www.eecs.qmul.ac.uk/mmv/datasets/deap/) and peripheral physiological signals was collected, while the participants watched 40 one-minute music videos [72]. A dataset for studying social stress using blood volume pulse (BVP) and electrodermal activity (EDA) signals has been recently published [98]. Cognitive load, effect, and stress recognition have been studied in [99] through recording the biosignals (ECG, PPG, EDA, and accelerometer data) of 62 healthy volunteers while answering math problems, logic problems, and the Stroop test. The Stanford wearable dataset (http://ipop-data.stanford.edu/wearable_data/Stanford_Wearables_data.tar) was used in [9] for arrhythmia detection and classification.

## 3. Challenges for ML Applications on Wearable Devices

Developing machine learning applications in general follows the Cross-Industry Standard Process for Data Mining Cycle (CRISP-DM 1999) [100]. The development-to-deployment process involves many challenges in collecting the data, selecting the best features, selecting the libraries and framework [100], evaluating the trained model(s), selecting the best model, and relying on the ML model decision since practically no ML model is guaranteed to be 100% accurate. ML learning models for health care are to be designed to generalize well and deal with unseen examples while taking into account personal features, providing interpretation for the result, and communicating the results cautiously. Some issues can be handled through clinical and preclinical studies, to provide a suitable user interface and a note for confidence or reliance on the results to be provided as per the regulatory requirements. The model needs to be implemented and used in both retrospective and prospective studies, and the clinical impact measured [101].

In addition to the typical challenges facing any machine learning application concerning the used data and model, there are many challenges that developers of a machine learning application for a wearable device should take care of, all challenges are shown in Figure 5 and are presented in the next subsections, and how they affect the choices available for developers.

### 3.1. Data Availability and Reliability

Machine learning approaches, in general, and especially in certain healthcare applications, require the availability of enough data for training to generalize well for unseen data. As presented in Tables 1–3 in the last section, the study with the maximum number of subjects [9] included 53,877 patients in a retrospective study that was funded by a commercial company for manufacturing ECG patches. The rest of the studies depend on far fewer data since the health data collection is expensive, which makes their results questionable for reliability.

The data obtained from wearable technologies have to be reliable as well with definite confidence and clear warnings to ask for medical staff help for any concern as human health is the ultimate goal. The authors in [102] investigated the sources of inaccuracy in different wearable optical heart rate sensors. They explored heart rate and PPG data from consumer and research-grade wearables while doing different activities for different skin tone subjects. According to their findings, there was statistically no significant difference in accuracy across skin tones, but significant differences between devices and between activity types were remarkable with an average absolute error of 30% more than during rest. The reliability of data in health care is so important for the patient and physician to rely on the device readings to take the most appropriate medical decision, which may in some cases threaten the life of a human. This what led Verily Life Sciences (formerly Google) to discontinue their glucose-sensing lens project (https://www.business-standard.com/article/news-ians/google-halts-project-to-build-glucose-sensing-contact-lens-118111800398_1.html) when their findings reveal that there is insufficient consistency in the correlation between tear glucose and blood glucose concentrations. Theranos is another example that went dreadful after being charged for wire fraud (https://www.fda.gov/inspections-compliance-enforcement-and-criminal-investigations/press-releases/june-15-2018-theranos-founder-and-former-chief-operating-officer-charged-alleged-wire-fraud-schemes) when investigations found they advertised rapid blood test devices that they knew were likely to contain inaccurate and unreliable results for different blood tests.

To ensure data reliability, conducting a wide range of clinical experiments while reporting the results transparently is critical for evaluating different techniques [103] and finding promising research directions. Medicolegal aspects need to be well-defined and regulated [104]. As an example, the authors in [105] provide guidelines for future study data collection and design for heart rate data, data cleaning and processing, analysis, and reporting that may help alleviate the data reliability challenge.

### 3.2. Model Selection and Reliability

For reliably calculating the accuracy of machine learning models, the use of cross-validation techniques is considered one approach to achieve this by testing the model on unseen data that have not been used in training. In [106], the authors reviewed the research work of using either record-wise or subject-wise cross-validation. They experimented with a publicly available dataset for activity recognition and simulation data to find that using record-wise cross-validation overestimates the prediction accuracy of machine learning algorithms. This result agrees with the research findings in [27]. Differently, some of the authors in [107] criticized the work done in [106] with arguments that no within-subject dependence between observations can be detected so record-wise cross-validation can be used. The authors also suggest avoiding leave-one-out cross-validation and recommend keeping the number of folds large enough while following strategies such as repeated test-train split, shuffle-split, repeated K-fold, or Monte Carlo cross-validation to avoid overfitting and ensure generalization. For wearable devices, since the models usually represent.

For model selection, there are many criteria that affect the decision when it comes to wearable devices [43]. One of them is to maximize the evaluation metric used to report accuracy for classification or minimize the error metric used in regression problems. Usually training an ensemble of different models achieves the best performance. Interpretability or explainability of the model [108] is another criterion as most of the applications for wearable devices target healthcare application for which the result of classification/regression or clustering is to be explainable and makes sense for the user. Tree-based models are seen as more interpretable than neural network-based models [43]. The size of the model to fit on the wearable device with limited memory is among the criteria. Additionally, the computational complexity for inference and for online training on the device for personalization is a concern due to the limited computation power for wearable devices until now. On-device deep learning and transfer learning for personalization have been researched in [43, 109–111].

### 3.3. Deployment Alternatives

There are three deployment alternatives for the machine learning model for the wearable device scenario, either to deploy the model on the wearable device, or on an edge device or on the cloud as shown in Figure 1. Each deployment alternative has some advantages and disadvantages that might make it impractical in some cases. Deploying the machine learning model on the device has the advantages of keeping the data private and decreasing the latency for the prediction/classification as there is no need to transmit large amounts of data from the device to the cloud. In particular, for healthcare applications, having the patient's data and the machine learning model on the device is more safe from privacy-preserving perspective. Low-latency and real-time feedback is also required for many healthcare applications that require immediate alert for the users or their caregivers such as fall detection and stress detection. On the other side, the main disadvantages of on-device computing include the limited device computing power, storage, and battery life.

With these limitations, offloading computations to be done on one or more edge devices (e.g., smartphones or locally on a hospital/house/office terminal/gateway) is one solution [112]. Edge/fog computing has also many advantages over the cloud computing alternative [112] in terms of security, latency, power consumption, real-time processing, and bandwidth load [113]. Edge computing can reduce data transmission to the cloud and consequently reduce power consumption and improve privacy by analyzing sensitive private data on a local gateway, filtering it, and compressing it, instead of doing it on a cloud away from the user's control. However, this depends on the size of the machine learning model and the data streams to be used in training and testing, the need for online training and real-time prediction, and the computational power needed for training and testing.

The main advantage of adopting cloud computing is the flexibility of storage and computational resource on-demand scalability. This comes as a trade-off for higher costs, power consumption, latency, and challenges for preserving the privacy of both the data and the machine learning model as will be discussed later.

Data drift (how data distribution could change over time) and continuous integration and delivery are other aspects that determine the decision of which deployment alternative to employ in machine learning applications for wearable devices.

The development process for wearable machine learning-based software requires the same operations for any software with some specific operations related to machine learning applications such as data collection, cleaning and preprocessing, continuous (re)training of the ML model, and continuous (re)-deployment of the updated model to the device or to the edge nodes or to the cloud service [114].  Figure 6 shows the typical machine learning operations (MLOps) in the development process of wearable software for ML-based applications with the different deployment alternatives (device, edge node, cloud service). The feedback arrows from the deployment process are orchestrated based on the performance of the model on edge nodes or cloud service after getting feedback from users or updated models received in case of federated learning scenario, which will be discussed in Section 3.8.3 to ensure continuous integration (CI) and continuous deployment (CD) requirements. Tools such as Apache Airflow, Kubeflow, and Google Cloud AutoML support the software lifecycle operations of ML components by orchestrating the different deployment alternatives and maintaining the continuous update of the ML cycle. A survey for the different automated machine learning approaches to automate feature extraction and selection, hyperparameter optimization, pipeline optimizers, and neural architecture search for healthcare systems can be found in [115].

### 3.4. Power Consumption

Power consumption is the main limitation of wearable devices due to their limited battery lifetime in general. For machine learning applications on wearable devices, the power consumption is greatly affected by the need to send physiological data measured by the device's sensors to the cloud to perform computations on the cloud. At the time of writing this study, the best commercial smart watch battery lifetime is just a few weeks, which monitors walking and running activities and give an approximate measure of the pulse rate and oxygen saturation. This could be far less in practice and could be as low as a few hours for wearables that monitor multiple vital signs continuously for alerting users to abnormal situations (e.g., alerting for abnormal heart rhythm or detecting fall).

The elements that affect the power consumption in wearable devices include the board, its components of different biosensors and their sampling rate, the operating system and other software running on the board, the wearable display, the rate of logging data on the device, and the amount of data transmitted over the communication channel (e.g., Bluetooth or Wi-Fi) to be sent to the edge/cloud.

Transmission and reception of data are thought to consume more energy than sensing and logging data. Research in the area of reduction in the power consumption can be seen to go in different directions, developing special embedded hardware for running machine learning algorithms [116, 117], reducing data to be transferred [118–120], compression [121] or scheduling of the data to be transferred [122], computational offloading [123, 124], and developing self-powered wearable devices [125, 126].

One approach suggested by the authors in [127] to save the consumed power by the data transfer over the wireless connection is to perform embedded machine learning on the device, i.e., following the tinyML approach. According to the analysis in their work, this can increase the battery lifetime by more than 70%. Researchers in [128] proposed a hybrid approach of using less battery, low sampling rate, and wearable RFID tags, which can be powered intermittently by a reader with additional passive RF tags that capture the presence and use of specific objects for daily activities' recognition.

As previously mentioned, another way to reduce power consumption is to reduce the data stored and transmitted to the cloud, and the authors in [129] proposed a variant of symbolic aggregation approximation (SAX) tested for compressing heart rate data, which proved to achieve the best trade-off between different performance metrics for systems that require short latency.

### 3.5. Storage and Memory

Typically, existing wearable devices have limited memories (e.g., Apple Watch Series 6 released in September 2020 has only 1 GB RAM) due to small device size and weight requirements. Wearable and IoT devices use nonvolatile memory (e.g., flash, EEPROM, MRAM, and F-RAM) to ensure resilient system recovery on sudden shutdown with the limited battery lifetime and to ensure short boot time. While flash-based storage is considered a de facto storage standard for IoT devices for its speed and stability [130], F-RAM is commonly used for medical wearables for its low power operation and high-write cycle endurance, which allow it to reliably and efficiently store more data logs from sensors [129]. EEPROM is sometimes also used since it is more reliable and smaller than flash memories for applications that do not require frequent write operations and requires less power. In [131], the authors proposed using battery-backed RAM on wearable devices and efficiently offload energy-intensive tasks to the smartphone/edge device to perform small and energy-efficient tasks locally using battery-backed RAM.

In addition to the development of memory architectures (in-memory computing) and hardware (application-specific integrated circuits (ASICs)) that are capable of running machine learning applications on battery-operated devices, tinyML Foundation (https://www.tinyml.org/), which started in 2019, has also focused on significant progress on algorithms, networks, and models down to 100 kB and below to perform on-device analytics at extremely low power, thus minimizing bandwidth and latency concerns while providing higher privacy.

The practicality of deploying a machine learning application on a wearable device or an edge device depends on many factors: the size of the device, the data size (features and time span of physiological data used for prediction), the complexity of the model (no. of parameters and layers), and use of batch or real-time processing. A model with high accuracy often requires more memory for the number of parameters and layers in the model than lower accuracy models. Depending on the machine learning application, some machine learning models can reach up to an order of 100 megabytes or even gigabyte (specifically those including image inputs), which cannot fit on the best wearable device along with the memory needed for doing the computations.

Thus, research goes on in many directions to overcome these factors. From the data perspective, data selection and dimensionality reduction techniques are employed. From the model perspective, designing new models with acceptable prediction accuracy while minimizing model size and prediction costs such as Bonsai [132] is another approach. Compression of models can take place by pruning (using less number of weights), quantization (using less bits per weight) [133], and encoding. The authors in [134] reviewed model compression techniques. Some of these techniques are implemented in TensorFlow Lite (https://www.tensorflow.org/lite).

### 3.6. Utility and User Acceptance

Users of wearable devices have been growing over the past few years, especially fitness trackers. Nevertheless, there is still a lack of user acceptance to adopt other wearable devices incorporating AI solutions for healthcare tasks.

According to [135], 35% of 1,183 adult patients in France would refuse using wearable monitoring devices and AI-based tools in their care. Another study in the United States [136] examined the response of 307 consumers to the perceived benefits and risks of AI medical devices with clinical decision support (CDS) features. The results of the study show that performance/accuracy and communication, besides the ethical and regulatory concerns to keep the data private and secure, significantly contribute to the perceived risks of using AI applications in health care. Regulatory agencies should establish a standard and evaluation guidelines for the implementation and use of AI in health care. Privacy and security concerns are among the major concerns raised for the use of wearables. For example, there are security concerns raised for using Google Glass for recording people data without their permission. It has been proven to be a serious issue since it can be used (like any recording device) to steal passwords by recording and analyzing the shadows of finger movements on a screen while typing a password [137]. Thus, the first version of Google Glass failed to gain social acceptance [138] before releasing its second version and funding some research studies about its usability, for example, its desirability for a sample of school children with autism [139].

Another important factor for user acceptance is how comfortable the device is for daily use. Design guidelines for wearable devices are identified in [140]. For example, designing a wearable should follow the anatomical structure of the body, take into consideration different gender requirements, and choose materials that are comfortable for the body and do not cause irritation to the skin. Additionally, it is preferable to be used in a free-moving environment and it is required to be as easy as possible to use without the need for many setup and configuration steps. Thus, a wearable device should be compact and simple to operate and maintain while providing secure and private experience for both the wearer and the people around him. More awareness endeavors of the wearable technology to the public need to take place and the advertisers should abide by honest marketing about the product's actual impact.

### 3.7. Communication

In case of edge computing model, the intra-communication between the wearable device and the edge device can be done over one of the standards such as Bluetooth, Zigbee, RFID, NFC, and UWB. Usually, lightweight Bluetooth is employed for its low power consumption [141]. However, according to Bluetooth 5 specification, the Bluetooth protocol allows up to 7 devices' simultaneous connections to a device and practically performance degrades and pairing problems arise when there are multiple connections to a smartphone. Other factors that affect the choice of communication technology are the maximum distance between the wearable and the edge device, the required data rate for the wearable-to-edge device, and the required latency [142]. The intercommunications in the wearable model over the Internet run between the edge device and the remote service or directly between the wearable device and the remote service are two-way data communication channels over transmission control protocol (TCP) or user datagram protocol (UDP) at the transport layer with the Internet protocol (IP) at the network level. TCP/IP is mostly adopted for lossless transmission of health data or machine learning model parameters over wide area network (WAN).

At the application layer, hypertext transfer protocol (HTTP) is commonly used as the request-response model from the edge to the cloud services. TLS is often employed to secure HTTP communication over TCP; however, HTTP is resource-intensive and is more suitable to be used for edge or fog devices with high power and storage capabilities. Other less-weight application layer protocols include constrained application protocol (CoAP), message queuing telemetry transfer (MQTT), and advanced message queuing protocol (AMQP) [143]. MQTT is a well-known publish-subscribe model standard used for IoT and wearable devices for being a lightweight protocol. It can facilitate one-to-many communications between wearable device(s) with low power and storage and the edge device on the other side.

The two communication channels with their running protocols at different network layers are susceptible to the different well-known network security attacks.

### 3.8. Security and Privacy

User data captured on wearable devices and sent to machine learning cloud services as shown in Figure 1 are subject to many security and privacy threats [144]. For example, accelerometer and gyroscope data on a smart watch can be analyzed to reveal passwords and credit card information (https://securelist.com/trojan-watch/85376/). Other attacks on IoMT devices can be life-threatening such as attacks disrupting the medical service, e.g., denial-of-service attacks (DoS) and ransomware attacks. Whether wearable devices are used for health monitoring or for fitness tracking, sensors' data and other personal data are being exchanged and analyzed by machine learning services to detect patterns and do classification/prediction based on the data. While it seems to be “a no problem to share” for some users, most end users are skeptical about how their personal data exchanged with such services is being used and how secure they are against different types of attacks. The issue of security and privacy of personally identifiable information and medical data in wearable and other IoMT devices' applications is critical and is regulated by different data protection standards across the globe.

In the case of wearables, the connection is usually done over lightweight Bluetooth as mentioned earlier and as shown in Figure 1. Security guidelines for Bluetooth provided in [145] consider wearable sensor devices as “Class 1.5 Low Energy” devices with a maximum output power of 10 mW that can operate for up to 30 meters distance but are typically used within 5 meters. The guidelines show that for this class, each service request can have its own security requirements. It recommends the use of Security Mode 1 Level 4 for medical devices, which requires low energy secure connections authenticated pairing and encryption using AES-CMAC and P-256 elliptic curve to the edge device.

The main challenge for edge computing is to incorporate security into the design of wearable devices through using encryption and providing solutions to manage, update, and secure the wearable devices. Security risks include but are not limited to malicious hardware or software injections, denial-of-service attacks, and different routing and physical attacks. Some of these attacks can be defended using appropriate administrative policy settings and incorporating different ML-based solutions for detecting different attacks that may compromise the communication network, computations, battery consumption, or storage [146].

Additionally, securing the data stored on the cloud, which is fed to the machine learning inference model, and securing the model itself represent a big challenge [147]. Not only the medical data itself and the machine learning model are considered prone to privacy attacks, but also the social dynamics and interactions with other users can be analyzed as done in [148].

Potential solutions for privacy-preserving ML are discussed in detail in [149, 150]. These include techniques for achieving differential privacy, cryptographic techniques, and client-based federated learning techniques. The following provides a brief discussion of these methods.

#### 3.8.1. Differential Privacy

The differential privacy concept was first introduced in [151] and refers to the process of protecting private data by adding noise based on Laplace, exponential, or Gaussian distributions. The noise is added in such a way that enables data analytics while providing privacy guarantees of the perturbed data. Differential privacy can be useful for applications such as health care due to its useful properties such as group privacy, composition, and robustness to auxiliary information. With differential privacy, healthcare applications that employ machine learning algorithms can still learn from the distribution of data without revealing the actual data of the patients. However, researchers in [152] concluded that privacy compromises must be made to preserve utility, especially in the challenging multi-class classification tasks based on their experiments on two datasets with membership attack and attribute inference attack. This utility-privacy trade-off has also been discussed in [153], where the authors found that as the privacy level increases, the machine learning algorithm—differentially private stochastic gradient descent in their case—targets the body of the distribution but loses important information about minority classes such as dying patients and minority ethnicity that are usually represented in the tail of distributions.

Another challenge for practically using differential privacy in healthcare wearable applications is that it is best used for high-dimensional balanced big datasets. This is not the case in some personalized healthcare wearable applications such as a fall detector, which only learns from accelerometer signals where falls are considered of low frequency.

#### 3.8.2. Cryptography-Based Methods

Traditional cryptography is valuable and efficient to achieve confidentiality when used in secure communication between parties and outsourcing the data for storage, but it is not valid when we need to perform the computation on confidential data as it needs preliminary data decryption. Here, we introduce some methods employed to perform computations on sensitive data without violating privacy.

(1) Homomorphic Encryption (HE): the idea behind HE is to use special encryption functions that enable the computation of encrypted data [154]. HE ensures that the result from performing operations on encrypted data, when it gets decrypted, is equivalent to the result of performing the same operations without any encryption. HE has the drawback of being impractically slow. However, it has been getting more practical and standardized over the last few years. HE can play a very useful role in healthcare applications where privacy is crucial, and using the data is subject to regulations. Many works in literature have demonstrated the idea of using homomorphic encryption for privacy-preserving machine learning in medical applications [155]. Research studies in [156–161] have presented different techniques to train a logistic regression model over encrypted data using homomorphic encryption. In [162–164], techniques of using the naive Bayes classifier model without leaking privacy information by applying homomorphic encryption have been presented. Cheon et al. [165] have presented a technique to use a clustering model over encrypted data. They employed the mean-shift algorithm and homomorphic encryption for the arithmetic of approximate numbers. To overcome the computational load of the mean-shift algorithm, they performed each iteration on a sample of the data instead of the whole dataset.
(2) Trusted Execution Environments (TEEs): TEE is a secure area located inside the main processor in particular architectures. It ensures the confidentiality and integrity of the data and code within the TEE. Examples of TEEs are Software Guard Extensions (SGX) from Intel and TrustZone from Arm. Intel's SGX provides a trusted execution environment, called an enclave, which trusts only the CPU and the on-chip cache [166]. A user program (code and data) must be partitioned into an untrusted portion and a trusted portion that will run inside the enclave. SGX protects the confidentiality and integrity of code and data during execution within the enclave from malicious programs that may be running alongside it, including privileged programs, such as the OS and hypervisor. Hunt et al. [167] employed the SGX to build their system for privacy-preserving outsourced machine learning called Chiron to protect the training algorithm and the user data. Segarra et al. [168] employed SGX to present a secure streaming processing system specifically fitted for medical data.
(3) Secure Multiparty Computation (SMPC): SMPC offers cryptographic protocols in which the computation is distributed across multiple parties where no individual party can see the other parties' data [169]. Two common approaches to achieve SMPC are garbled circuits and secret sharing.
  - Garbled Circuits: in this technique, two (or more) parties can jointly evaluate a function over their private inputs [170]. The main idea behind this technique is to use a Boolean circuit to represent the function that needs to be evaluated. The gates of the function are garbled by one party, and the private inputs are garbled and exchanged using an oblivious transfer protocol. A garbled circuit can provide a solution for privacy-preserving computations [171]. For example, consider a patient who wants to use a diagnosis service without revealing his data and a service provider also wants to hide his algorithm parameters, which are considered trade secrets. In this case, a service provider can convert his algorithm into a Boolean circuit, garble the circuit, and send it to the patient to be evaluated without loss of privacy.
  - Secret Sharing: in this technique, an entity can preserve the privacy of its sensitive data by breaking it up into multiple shares and distributing the shares to a set of non-colluding parties where each party computes a partial result depending on the shares it received [172]. Finally, one of the parties can receive these partial results and combine them to get the final result.

SMPC protocols are widely used to provide privacy-preserving in machine learning applications. However, SMPC fails to protect against exploratory attacks. Exploratory attacks act by performing several queries on a fully trained model to leak some information about the model parameters and its training data, such as if a specific example was used in the training set or not. With this information, the attacker can gradually train a substitute model that reproduces the same prediction of the target model [147]. To address these kinds of attacks, Kesarwani et al. [173] proposed a monitoring scheme called extraction monitor to track the queries issued by the user, evaluate the information that a user might leak from these queries, and give a warning when the user exceeds the average number of queries needed to reconstruct the model.

#### 3.8.3. Federated Learning Methods

Federated learning was first introduced in [174]. Federated learning is a machine learning setting in which many devices collaborate in training a model in a centralized manner while keeping the training data private and decentralized [175]. In the cross-device federated learning setting, the server sends out an initial model to the devices, and the clients then train the model on-device with their data locally and send the updated device model to the server. Updated models are combined at the server using federated averaging to update the initial model. This process goes on by sending the updated combined model until the metrics are satisfactory.

This approach was tested in [176] by applying federated learning to heart activity data collected from multiple smart bands in a stress-level monitoring scenario. The authors achieved comparable accuracy while preserving the privacy of the data and reducing the communication burden by only communicating the models' parameters. Additional privacy-preserving protections such as secure multiparty computation or differential privacy may further be included in the federated learning setting to keep data and model statistics private from malicious clients [177]. In the research done by [178], the authors utilized both SMC and differential privacy to balance the trade-off between vulnerability to inference and low accuracy in a federated learning setting.

For most of the healthcare applications, the machine learning model is better to be personalized as per the biosignals for each patient. Model aggregation with federated averaging as mentioned above does not provide this personalization. The authors in [179] applied transfer learning in the federated learning setting so that each device can train a personalized model tailored to the user's data by utilizing the cloud model and data and the local data.

## 4. Discussion

The use of artificial intelligence research has clearly been rapidly growing in healthcare applications. However, for healthcare wearable devices, it can be seen that practical artificial intelligence and machine learning still face some challenges in medical wearable devices as presented in this review. In this section, we will discuss briefly a summary for the main perceived pitfalls or difficulties facing applying machine learning research for wearable devices and highlight the related machine learning research directions that need further development.

The training data input to a machine learning model is considered the most crucial element in the machine learning process as garbage in mean garbage out. The first step is to choose well-calibrated sensors that are better validated against benchmarked devices used in hospitals that have undergone plenty of clinical experiments or other gold standard devices [180]. Care should be taken as some of the research wearable devices provide raw data [102] that require clean-up of the signals for removing noise and motion artifacts as the work done in [181]. Identifying the inaccuracies in the data collected and considering that most of the sensors are only accurate during rest [102] have to be taken into account as this has implications on the drawn conclusions and health-related decisions using wearable devices in research. Most of the research works that have been cited in Section 2 use research-grade wearable devices and do not mention the preprocessing and cleaning up steps of data. Signal processing techniques are better to be employed to cure these signals and remove motion artifacts [182]. Moreover, clinical experiments are to be done to help in defining the reference signal/ground truth and obtaining clinical evidence.

For some applications, the ground truth signal is not known due to the complexity of the human body's response and the different responses for each individual. For this reason, the collection of data from as many subjects as possible is recommended to develop algorithms to clean the data and build more accurate models that generalize well. However, the process of data collection is an expensive and time-taking process that most academic research work cited in Section 4, which was not funded by companies, depending on data from a relatively small set of subjects. A transparent and reproducible process for collection of data from wearables, training, and evaluation of models is recommended for gaining trust in the research results and effectively building over accumulating research efforts. The authors in [183] pointed out recommendations for reporting machine learning results in clinical research and similar guidelines are to be followed for machine learning research for wearable devices, especially those used in healthcare as they affect human life.

One cheap approach for big data collection is crowd-sourcing data collection such as the one initiated by a research group at Stanford University (https://innovations.stanford.edu/wearables), which collects data from wearable devices remotely through a mobile application. However, this approach is susceptible to many privacy issues that existing commercial smart watch entities do not handle and the data collection process will be only protected by the privacy policy of the application. Privacy-aware sharing of data and learning from it without revealing the actual users' data employing some privacy-preserving techniques mentioned in the last Section 3 is an active research area. An example for that is the work by the authors in [184] for privacy-preserving data collection using a local differential privacy technique over salient data to protect users' data. Research work in differential privacy has also open issues to investigate new learning solutions, which can learn from data distribution tails (data that represent minority class) effectively while maintaining an acceptable privacy loss as suggested by [153]. Federated learning is also a relatively new privacy-preserving method that needs further attention and exploration in the field of machine learning for wearable devices, which can also promote the personalization of the local model.

Another approach for augmenting the data input to the ML model is generating training data using generative adversarial network (GAN) variants that may help train good quality models without exposing users' wearable data and signals used in training or without even using any real data but only simulated data as in [185].

For guaranteeing some level of privacy for users of wearable devices, the machine learning application, which usually holds identifiable information at the edge device (e.g., smartphone running the application), should follow a set of regulations to gain users' trust. Besides compliance with HIPAA (Health Insurance Portability and Accountability Act: https://www.hhs.gov/hipaa/for-professionals/index.html), GDPR (General Data Protection Regulation: https://gdpr.eu/), HITECH (Health Information Technology for Economic and Clinical Health: https://www.hhs.gov/hipaa/for-professionals/special-topics/hitech-act-enforcement-interim-final-rule/index.html), and act regulations, machine learning applications for wearable devices should follow the OWASP security standards (Open Web Application Security Project (OWASP): https://owasp.org/www-project-top-ten/).

Among other data challenges in machine learning for wearables is identifying which data to be collected from these devices. Different modalities can increase the accuracy of the model as usually many signals can be used for a single task. Another big challenge is how to model the uncertainty arising from the complex input received by the human body as shown in Figure 2, which may affect the accuracy of any model. For example, considering the stress detection task is a complex task that involves many inputs and can affect many body systems. Using multimodal sources is believed to be a very rich source of information that can help in health monitoring by identifying the emotional state, stress level, and diagnosis of some diseases. As an example, monitoring audio signals from the user to detect laughing, crying, shouting, or coughing can help in these applications on wearables, but it faces other challenges [186]. EEG signal, despite the difficulty of capturing it, can also hold a lot of information, which can help in achieving higher accuracy in many applications such as dehydration detection, emotion recognition, and mental disorders detection.

Moreover, depending on learning from only few body signals, which may also be noisy, would lead to uncertain decision from the ML model. As handling and estimating uncertainty in ML modeling remain an active area of research in ML, we recommend applying its techniques in the wearable healthcare domain to give insight into the confidence in the ML model, which would be helpful, especially in tasks such as seizure detection and diseases' diagnosis devices. Besides uncertainty modeling in wearable ML applications, joining upregulation among key stakeholders in the field of healthcare wearables is a key to make sure that ML is introduced in wearables with more transparency from tech companies and for gaining better users' trust and acceptability. As it is pretty obvious, ML applications for healthcare wearables are a multidisciplinary field that requires standards about naming conventions, evaluation metrics, ethical reporting of research results, and clinical impact as suggested in [101] as these devices may directly affect human life. Mentioning evaluation of machine learning models, it was found that the use of subject-based cross-validation is recommended since subject data represent a clinically more relevant scenario for disease diagnosis application than using records from a subject in training while using some other records for the same subject in testing the machine learning algorithm. This can let the machine learning algorithm learn an association between unique features of the same subject and accordingly may fall into overfitting. This raises a question about whether building personalized models can be more effective as it learns from signals of the same individual to avoid averaging out important individual characteristics such as age, sex, weight, height, eating style, and way of doing an exercise [26]. Furthermore, personalized models can learn from much less data and guarantee better privacy for data.

Deciding upon the time window of the signal to learn from is yet another challenging decision as more data do not necessarily mean better results. It faces memory limitations on the wearable device and power limitations for sending this amount of sampled data from the device to the edge or to the cloud. Consequently, the sampling rate for different physiological signals needs to be optimized as per the application to optimize the use of resources and decrease the power consumption. Nevertheless, exploring tinyML embedded solutions and models' optimization techniques in IoT is a recent research area that is open to some applications in healthcare wearables as well. However, for computationally intensive applications, full computation offloading can be effective while for data-intensive applications offloading techniques that offload the processing of some of the data will be more suitable as suggested by [187] while preserving the privacy of users' data.

Most of the research works for applying machine learning for healthcare wearable devices tasks that we reviewed in Section 3 are experiments for learning from data obtained from one or more sensors for detection or recognition of some pattern. Complete analysis of the proposed models in terms of memory requirements and amount of communicated data in case of edge or cloud deployment, which greatly affects power consumption, is better to be provided.

Overcoming these difficulties with AI solutions, together with the ongoing research and development in the field of medical sensors, storage, SoCs, and power-efficient management and generation for wearable devices, would ensure having AI-enabled healthcare wearable devices that can help reliably with remote patient monitoring, detect problems with the human body earlier and assist in diagnosis, perform elderly people care and monitoring, and act as a lifestyle guide and much more. A lot of many other AI applications can receive user acceptance by solving problems with the reliability, comfort, and privacy of the wearable devices.

## 5. Conclusion

The growth of using wearable devices over the recent years is clearly noticeable. With the huge amount of research efforts to employ artificial intelligence solutions in healthcare-related tasks for wearable devices, their use is expected to grow even more and change from a “nice to have” devices with fun applications to necessary devices for remote patient monitoring and detection of any irregularities with the human body. In this review, we presented ML tasks that have been researched in the healthcare wearable devices field, the machine learning techniques used, the different modalities used, and the available datasets in the field. The different challenges facing machine learning applications on wearable devices (deployment alternatives, power consumption, storage and memory, utility and user acceptance, data availability and reliability, communication, security and privacy) were discussed while identifying possible solutions found in the literature. Finally, the study highlights issues that require further research concerning data availability, reliability, and privacy to enable effective and efficient learning from data generated by wearable devices.

Contents of the research are solely the responsibility of the authors and do not necessarily represent the official views of the Qatar National Research Fund (QNRF).

## Figures and Tables

**Figure 1:** Wearable device application model.

**Figure 2:** Human body as a system and signals that can be used as a source of data for machine learning models.

**Figure 3:** Healthcare machine learning tasks and sensors used for each one in literature.

**Figure 4:** Box plot of accuracy for the machine learning techniques used in different classification problems for papers cited in Tables 1–3 with accuracy as the evaluation metric. On each box, the central mark is the median and the edges of the box are the 25th and 75th percentiles. The small circles represent outliers.

**Figure 5:** Challenges to healthcare ML applications on wearable devices.

**Figure 6:** MLOps for wearable device application.

**Table 1:** Machine learning research work for healthcare wearables for fall detection, activity recognition, eating monitoring, fitness tracking, and stress detection.

Task	Research work	ML technique(s)	Sensors/signals used	Dataset(s)

Fall detection	[48]	J48 (96.7%), logistic regression (94.9%), MLP (98.2%)	3D accelerometer and gyroscope in smartphone	MobiAct (https://bmi.hmu.gr/the-mobifall-and-mobiact-datasets-2/)
	[49]	KNN (84.1), naive Bayes (61.5%), SVM (68.25%), and ANN (72%)	Accelerometer, gyroscope, and magnetometer	UMAFall dataset (https://figshare.com/articles/dataset/UMA_ADL_FALL_Dataset_zip/4214283)
	[30]	Temporal signal angle measurements	Inertial measurement unit (IMU)	12 features for 7 subjects performing 5 fall types
		(93.3%@200 Hz to 91.8%@10 Hz)		(9 times each with 3 different speeds)
	[50]	KNN and RF	Accelerometer and gyroscope	SisFall dataset [51]
		(99.80% KNN and 96.82% for falling activity recognition)		(For falling and non-falling activities)
	[52]	SVM (97% F1 score and 99.7% recall)	Accelerometer and gyroscope	Public fall detection dataset [27]

Activity recognition	[25]	CNN	Accelerometer and gyroscope	UCI-HAR dataset and study set
		(UCI-HAR dataset: 95.99%, study set: 93.77%)		21 participants and 6 ADLs
	[53]	Locally linear embedding transfer learning	Accelerometer, magnetometer, gyroscope	UCI-HAR dataset
	[26]	Sequence-to-sequence matching network	Tri-axis accelerometer, tri-axis gyroscopes, magnetometer (depending on the dataset)	Postures dataset, mini MobiAct, and UCI-HAR dataset
	[54]	SVM: 90%	sEMG signals of the upper limb by Delsys, accelerometer	6 males and 6 females for 3 motion states of virtual vehicle: left turn, stop, and right turn
	[39]	ATRCNN: 97%	Tri-axis accelerometer, tri-axis gyroscope	6550 pieces of data for 4 activities: walking, sitting down, running, and climbing stairs

Eating monitoring	[34]	Proximity-based active learning	3D accelerometer	A public dataset for performing different activities including eating [34]
	[55]	Random forest (89.6% in the laboratory and 72.2% outside the laboratory)	One IMU and a proximity sensor on ear and one IMU on the upper back and a microphone	Two datasets: 12.5 hrs for 16 participants in semi-controlled setting with 6 labels and 3 hrs for each of 15 participants outside the laboratory with chewing and non-chewing labels
	[37]	DBSCAN clustering	3D accelerometer	A public dataset for performing different activities including eating [34]
	[56]	Random forest and DBSCAN clustering algorithm (average precision of 92.3%)	Inertial sensor on the downside of the lower jaw	A study dataset of 25 participants, 10 in a laboratory setting and 15 in the wild doing different activities including eating a meal of different food types
	[33]	Gradient boosted decision tree (80.27% accuracy)	Gyroscope and accelerometer in Apple Watch	79 features for 16 subjects taking pills

Fitness tracking	[38]	Logistic regression (0.9356), random forest (0.9203), extremely randomized trees (ERT) (0.9177), and SVM (0.9328)—best accuracy reported in different scenarios	2 accelerometers (hip and ankle)	Study set of 39 participants with a total of 55 days in which sport and jogging activities were logged
	[57]	L2-SVM	3-Axis accelerometer and 3-axis gyroscope	114 participants over 146 sessions

Stress detection	[2]	BN, SVM, KNN, J48,	Zephyr BioHarness for ECG	2 participants with 324 instances
		RF and AB learning methods	Shimmer3 GSR for EDA	At rest and exercise sessions
	[24]	Neural network model (92% accuracy for metabolic syndrome patients and 89% for the rest)	ECG, GSR, body temperature, SpO2, glucose level, and blood pressure	312 biosignal records from 30 participants
	[58]	LR (87% accuracy) and SVM (93%)	ECG sensor in a chest strap	HR and RR data for 44 children (26 with ASD and 18 without ASD) while at rest (7 min) and while engaged in stressful tasks (9 min)

**Table 2:** Machine learning research work for healthcare wearables for arrhythmia detection, seizure detection, rehabilitation tasks, and hydration monitoring.

Task	Research work	Techniques	Sensors	Dataset(s)

Arrhythmia detection	[59]	SVM and K-medoids clustering-based template learning	ECG and PPG sensors	14 subjects recordings for a 30-minute training session and a 30-minute testing session
	[60]	Deep learning (max 89% accuracy)	ECG sensor, PPG sensor (SpO2)	Cleveland database on UCI
	[9]	DNN (0.837 F1 score)	ECG patch (from iRhythm)	91,232 single-lead ECGs from 53,549 patients
	[61]	50-Layer convolutional network (95% AUC)	PPG sensor	402 PPG recordings for 29 free-moving subjects (13 with persistent AF) and the NSR dataset of 341 PPG recordings from 53 healthy free-moving subjects
	[10]	Deep learning (94.7%)	PPG sensor in a ring-type device	13,038 30-s PPG samples (5850 for SR and 7188 for AF)
	[11]	SVM and bagging trees	ECG	Public available dataset from Computing in Cardiology Challenge (CinC) 2017 (https://physionet.org/content/challenge-2017/1.0.0/)
	[4]	ResNet of 34 layers of 1D rectified linear unit	Acoustic recordings	5878 deidentified audio recordings, totaling >rbin 34 hours from 5318 unique patients labeled by a majority vote of 3 cardiologists as heart murmur, no heart murmur, or inadequate signal

Seizure detection	[62]	SVM (97.31), RF (97.08), NB (95.08), K-nearest neighbor (90.01), and neural network (93.53)	EEG	UCI EEG sampled dataset for epileptic seizures
	[63]	SVM ((Sens > 92%) and bearable FAR (0.2–1))	Accelerometer and electrodermal activity from Empatica Embrace	135 patients with generalized tonic-clonic seizures with 22 seizures
	[64]	Not mentioned	Accelerometer and electrodermal activity	40 pediatric patients with generalized tonic-clonic seizures
	[65]	Two classifiers (the models are	EDA and accelerometer	5,928 h of data of 55 convulsive
		not mentioned) best sensitivity 95% and < 1 false alarm rate	from three wristbands	Epileptic seizures from 22 patients
	[8]	LSTM and 1DConv	Temperature, accelerometer	69 patients with epilepsy
			Blood volume and EDA	(total duration > 2311 hours, 452 seizures)

Rehabilitation tasks	[66]	SVM, RF	sEMG acquisition module	Muscle signals sEMG for 3 users doing 9 hand gestures 12 times
	[67]	K-means clustering, SVM, and artificial neural network (ANN)	IMU sensor module and plantar pressure measuring foot insoles	81654 samples for 10 people data, each sample has 10 features calculated from 64 sensing nodes in the foot insole
	[68]	Support vector regression (SVR)	IMU in SportSole	Inertial features and anthropometric characteristics of 14 healthy subjects
	[69]	Multiple regression, inference tree, and RF	Two-sensor (fore and aft) insole (LoadsolTM)	Kinematic and pressure features for 30 participants, each doing 120 steps

Hydration monitoring	[70]	SVM for drinking detection	Acoustic sensor	Frequency and cepstral domain
		Gradient boosting decision tree for activity recognition	and inertial sensor	Features are extracted from the signals
	[21]	LDA, quadratic discriminant analysis, logistic regression, SVM, Gaussian kernel, KNN, decision trees, ensemble of KNN	EDA and PPG	51 hydrated samples and 17 dehydrated for 17 subjects with features from EDA and PPG
	[71]	SVM (60%) and K-means clustering (42%)	ECG (not wearable (RR interval, RMSSD, and SDRR recorded))	10 minutes ECG for 16 athletes at rest, post-exercise, and post-hydration
	[43]	DNN, RF, extra trees	Shimmer (IMU, GSR, PPG, etc.)	3386 min for 11 subjects under fasting and non-fasting conditions

**Table 3:** Machine learning research work for healthcare wearables for emotion recognition, sleep monitoring, and disease diagnosis.

Task	Research work	Techniques	Sensors	Dataset(s)

Emotion recognition	[16]	Liquid state machine (LSM)—above 94% accuracy for valence, arousal, and liking recognition	EEG sensor	DEAP dataset [72]
	[73]	KNN (accuracy ranges from 53.6% to 69.9%)	MUSE headband (EEG) and Shimmer GSR + device (SC and HR)	54 subjects watching 24 pictures
	[74]	Random forest, SVM, and logistic regression—73.08% for arousal and 72.18% for valence	Respiratory belt (RB), PPG, and fingertip temperature sensor	DEAP dataset [72]

Sleep monitoring	[1]	Auto-correlated wave detection with an adaptive threshold (ACAT), accuracy for UCI-HAR dataset: 95.99%, study set: 93.77%	Accelerometer and gyroscope	UCI-HAR dataset and study set of 21 participants and 6 ADLs
	[32]	Random forest (F1 score: 73.93%)	Accelerometer in wristband	Accelerometer data during one night for 134 participants (70 with sleep disorder and 64 good healthy sleepers)

Disease diagnosis	[75]	ResNet with LSTM for hypertension detection	ECG, PPG, and invasive BP in ICU	(MIMIC III) waveform database for ICU patients and a database of patients with cardiac arrhythmias collected from Fuwai Hospital, Chinese Academy of Medical Sciences
	[76]	Machine learning techniques for early detection of COVID-19	Everion wearable (skin temperature, respiratory rate, blood pressure, pulse rate, blood oxygen saturation, and daily activities)	200–1000 asymptomatic subjects with close COVID-19 contact under quarantine in Hong Kong
	[22]	Multivariate regression for case deterioration	Heart rate, heart rate variability, respiration rate, oxygen saturation, blood pulse wave, skin temperature, and actigraphy	34 patients with PCR-confirmed COVID-19 were admitted to the isolation wards of Queen Mary Hospital
